# Identification Method of Citrus Aurantium Diseases and Pests Based on Deep Convolutional Neural Network

**DOI:** 10.1155/2022/7012399

**Published:** 2022-05-27

**Authors:** Yuke Lin, Jin Xu, Ying Zhang

**Affiliations:** ^1^Department of Communication Engineering Chongqing College of Electronic Engineering, Chongqing 401331, China; ^2^Dabashan Branch of Chongqing Academy of Chinese Materia Medica, Chongqing 400065, China; ^3^Disinfection and Vector Control Institute of Chongqing Center for Disease Control and Prevention, Chongqing 400042, China

## Abstract

The traditional identification methods of Citrus aurantium diseases and pests are prone to convergence during the running process, resulting in low accuracy of identification. To this end, this study reviews the newest methods for the identification of Citrus aurantium diseases and pests based on a deep convolutional neural network (DCNN). The initial images of Citrus aurantium leaves are collected by hardware equipment and then preprocessed using the techniques of cropping, enhancement, and morphological transformation. By using the neural network to divide the disease spots of Citrus aurantium images, accurate recognition results are obtained through feature matching. The comparative experimental results show that, compared with the traditional recognition method, the recognition rate of the proposed method has increased by about 11.9%, indicating its better performance. The proposed method can overcome the interference of the external environment to a certain extent and can provide reference data for the prevention and control of Citrus aurantium diseases and pests.

## 1. Introduction

Citrus aurantium (bitter orange) is an herbal medicine collected in the Chinese Pharmacopoeia, and its medicinal source is the dried fruit of the Rutaceae plant lime and its cultivars. The green peel is harvested in July, cut in half from the middle, and dried in the sun or at a low temperature. Citrus aurantium is bitter, acrid, sour, and warm and has the functions of regulating qi and unblocking the stomach, promoting qi, and stopping bloating. It is mainly used to treat diseases such as qi stagnation in the chest, distending pain, undissolved food accumulation, phlegm-rheum collecting internally, gastroptosis, anus prolapse, uterine prolapse, etc. Citrus aurantium is produced in many places in China, mainly in Hunan and Jiangxi provinces. Specifically, Citrus aurantium from Xingan County, Jiangxi Province, is also known as Shangzhou Citrus aurantium and Sanhu Citrus aurantium, with the characteristics of thick pulp, eversion like raspberry, and many orange petals. Its medicinal ingredients are better than other varieties, and it is listed as a protected product of China's National Geographical Indication [1]. With the development of the Citrus aurantium industry, the variety of the diseases and pests of Citrus aurantium has increased and the degree of damage has worsened. It is urgently needed to find ways to quickly and accurately diagnose Citrus aurantium diseases and take corresponding control measures.

In terms of diseases and pests detection, the commonly used method is to manually identify with the naked eye by agricultural experts. This method can compare plant insect and pest samples based on external characteristics, such as shape, color, etc., to obtain identification results. However, because manual identification has certain limitations and subjectivity, and humans cannot continuously work for a long time, the accuracy of manual identification is low, and it is labor-intensive. This has led to the contradiction between the growing demand for identification of crop diseases and pests and the shortage of identification staff in China [2]. For this reason, researchers have put forward a method for the identification of Citrus aurantium pests by combining computer technology and image processing technology. So far, the research fields related to crop disease image recognition have made some progress and achieved many research results. The existing research results include the proposal of pest identification method based on deep learning [3], machine vision [4], and spatial pyramid pooling [5].

At present, most of the image features are extracted by artificial design or through spectral discrimination. However, the traditional identification methods of Citrus aurantium diseases and pests are prone to convergence during the running process, resulting in low accuracy of identification. Different environmental conditions have a great impact on the recognition results, and the robustness and accuracy are poor. To this end, this study introduces a DCNN algorithm. The DCNN algorithm is a combination of the deep learning algorithm and the convolutional neural network (CNN) algorithm, which solves the problem that the traditional CNN is prone to convergence and falls into local minimum points during the propagation process. In the DCNN algorithm, deep learning technology is used to automatically extract features of the images. The application of DCNN method to the identification of Citrus aurantium diseases and pests can improve the identification efficiency and provide effective technical support for the control of Citrus aurantium diseases and pests.

## 2. Experimental Materials and Methods

### 2.1. Acquiring the Images of Citrus Aurantium Diseases and Pests

Firstly, the test object of Citrus aurantium was selected. Then, under natural lighting conditions, CCD cameras were to collect the images of Citrus aurantium diseases and pests under three automatic exposure modes with image resolution of 2048 × 1536, 1600 × 1200, and 1024 × 768, respectively. The images were saved in the unity environment in the same format. The specific steps of acquiring the images of Citrus aurantium diseases and pests are shown in Figure 1.

The images of Citrus aurantium diseases and pests were collected in three time periods, morning, middle, and evening. The collection points are randomly and uniformly distributed in the specified area. The camera was made parallel as much as possible to the plane where the leaves of the Citrus aurantium were located to prevent obvious deformation [6].

### 2.2. Image Preprocessing

There is a certain degree of irrelevant image information in both healthy and diseased Citrus aurantium images. Image preprocessing is to enhance relevant information and eliminate irrelevant information to the greatest extent, thereby improving the reliability of image recognition.

The different sizes of the images are not conducive to the convolution operation in the subsequent network training, and the main information is located in the middle area of the image. Therefore, images should be cropped in batches before classification and identification, and a final image size of 256 × 256 in the middle area should be selected. While simplifying the dataset, the number of datasets should remain unchanged, and the information of major diseases should be retained.

Furthermore, the image is directly compressed or expanded into a deep convolutional network model, which requires a fixed input image size. The input format required by the ResNet network model is 224 × 224, and the input format required by the Inception-v3 network model is 299 × 299 [7].

Image enhancement techniques include grayscale, binarization, filtering, and smoothing, etc. The commonly used RGB image is subjected to weighting processing on the three components of *R*, *G*, and *B* and then used as grayscale value. The process can be expressed as

(1) $$\begin{array}{c} \text{Gray}=0.299R+\;0.587G+\;0.114B, \end{array}$$

where *R*, *G*, and *B* represent the three components of the color image of Citrus aurantium, respectively, and the calculation result is the gray value of the pixel. On this basis, all the pixels of the original image are calculated, and the grayscale processing result of the color image is obtained. Using the grayscale histogram of the image, the image is divided into objects and backgrounds using a threshold. The expression is as follows:

(2) $$\begin{array}{c} g\left(x,y\right)=\left\{\begin{array}{cc} 1, & f\left(x,y\right)>T,\\ 0, & f\left(x,y\right)\leq T, \end{array}\right. \end{array}$$

where *f*(*x*, *y*) is the pixel value of point *g*(*x*, *y*) and *T* is the global threshold of the segmented image. Then, the median filter algorithm is used to filter the images. The median filtering algorithm uses some neighborhood pixels around the pixel to be processed to form a region space, arranges the gray values of all pixels in the region space from small to large or from large to small into a series, and then uses the middle value in the series as the gray value of the center point, as shown by

(3) $$\begin{array}{c} g^{\prime }\left(i,j\right)=\text{Med}\left\{g\left(x,y\right),\left(x,y\right)\in S\right\}. \end{array}$$

A new image can be obtained by performing the same processing on each pixel in the image in sequence [8]. In equation (3), if there is an odd number of pixels in the field space *S*, then the gray value of the pixel in the middle after sorting is taken as the gray value of the center point; if there is an even number of pixels in the field space *S*, the gray value of the middle two pixels is used as the gray value of the center point.

#### 2.2.1. Multiple Morphological Transformation

 Mathematical morphology usually has four basic operations, namely, erosion, dilation, closing, and opening [9]. In this study, two transformation methods, i.e., erosion and dilation, are mainly used in processing the images of Citrus aurantium. The corrosion operation is to eliminate boundary points and shrink the boundary inward. Target area of the image of Citrus aurantium is set as the set *A* which is subjected to convolution operation with the kernel *B*. The processing results are as follows:

(4) $$\begin{array}{c} A\Theta B=\left\{x|{\left(B\right)}_{x}\subseteq A\right\}. \end{array}$$

Equation (4) shows that, after translating *B* by *x* pixels, its solution still exists in the set *A*; then it is said to be eroded by *A*. Corrosion is mainly manifested as image shrinkage. Furthermore, the role of dilation is to blend the surrounding environment into the target area, so that the boundary expands outward. The result of processing the set *A* expanded by the set *B* can be expressed as

(5) $$\begin{array}{c} A⊕B=\left\{x|\left[{\left(B\right)}_{x}\subseteq A\right]\neq \emptyset \right\}. \end{array}$$

When performing polymorphic transformation on an image, the operation of first eroding and then dilating is called the opening operation, which can eliminate the small noise inside the image and smooth the boundary of the object. The operation of first dilating and then eroding is called the closing operation, which can fill the small holes inside the image and smooth the boundaries of objects [9]. After many times of opening and closing operations on the image of Citrus aurantium, morphological transformation is performed on it.

#### 2.2.2. Image Normalization

The role of the normalization operation in probability theory is to present the statistical distribution of the sample, and the interval is normalized to [0, 1]; then the interval presents the coordinate distribution [10]. To this end, the *Z*-score method is used to normalize the disease image dataset into the [0, 1] interval to meet the data input requirements of the deep convolutional network model. Its mathematical expression is

(6) $$\begin{array}{c} y^{\prime }=\frac{y-\mu }{\sigma^{2}}, \end{array}$$

where *y* represents the disease image dataset, the initial *μ* represents the mean value of the Citrus aurantium disease and pest data, and the parameter *σ* represents the variance of the Citrus aurantium diseases and pests data.

### 2.3. Constructing a DCNN

A DCNN is divided into input layer, feature extraction layer, and output layer from the perspective of data flow [11]. From the structural point of view, the DCNN consists of one or more convolutional layers, pooling layers, and fully connected layers. The two-dimensional image is used as the direct input of the network, and the middle part of the network is alternately connected by convolutional layers and pooling layers. The output layer is usually composed of a fully connected layer and a classifier, and the constructed DCNN structure is shown in Figure 2.

As can be seen from Figure 2, the DCNN consists of three convolutional layers, two pooling layers, and two fully connected layers. The size of the handwritten digit image input is 32 × 32. In the feature extraction layer, the convolutional layer receives the feature map of the previous layer and affines the convolution of the previous layer with the current layer [12]. The result of the operation is calculated, and the feature map of the layer is obtained through the activation function.

(7) $$\begin{array}{c} \left\{\begin{array}{c} y_{j}^{m}=f\left(u_{j}^{m}\right),\\ u_{j}^{m}=\sum_{i\in M_{j}}x_{j}^{m}*k_{ij}^{m}+b_{j}^{m}, \end{array}\right. \end{array}$$

where *y*_*j*_^*m*^ and *u*_*j*_^*m*^ represent the feature map and net activation of the *j* th convolution kernel of the *m* th convolution layer, *b*_*j*_^*m*^ represents the bias parameter, *k*_*ij*_^*m*^ represents the weight of the *j* th convolution kernel of the *m* th layer, and *f*(·) and *∗* represent the nonlinear activation functions and convolution operator, respectively. The downsampling layer of the DCNN performs aggregation statistics on the upper-layer feature maps through local correlation. By reducing the feature dimension, the signal-to-noise ratio can be improved, and local features can be fused to generate new features [13]. The downsampling extraction of the input feature map can be expressed as

(8) $$\begin{array}{c} \left\{\begin{array}{c} y_{j}^{m}=f\left(u_{j}^{m}\right),\\ u_{j}^{m}=\beta_{j}^{m}\text{ down }\left(x_{j}^{m-1}\right)+b_{j}^{m}, \end{array}\right. \end{array}$$

where down(·) represents the downsampling function and *β*_*j*_^*m*^ represents the weight of the *j* th convolution kernel of the *m* th downsampling layer. By rasterizing the input pixel values, the two-dimensional feature map is converted into a one-dimensional feature column, and then the output feature map of the fully connected layer is obtained by weighted summation and nonlinear activation function operation:

(9) $$\begin{array}{c} u^{m}=\omega^{m}x_{j}^{m-1}+b_{j}^{m}, \end{array}$$

where *ω*^*m*^ represents the weight parameter of the fully connected layer. To improve the recognition accuracy or meet the needs of specific tasks, multiple auxiliary layers such as dropout, local response normalization, local contrast normalization, and linear activation units are also inserted into the hidden layer in this study [14]. The activation function in the DCNN selects the sigmoid function which has the characteristics of monotonically increasing and inverse functions and can map variables to [0, 1]. The sigmoid function expression is given by

(10) $$\begin{array}{c} \text{Sigmoid}\left(\alpha \right)=\frac{1}{\left(1+e^{-\alpha }\right)}. \end{array}$$

The image corresponding to the sigmoid function is shown in Figure 3.

### 2.4. Segmentation of the Image Area of Citrus Aurantium Disease Spots

For the Citrus aurantium image, in the context of DCNN, HSI is selected as the color space. Among them, the I component has nothing to do with the color information of the image, while the H and S components are closely related to people's perception of color. Based on this feature, when H belongs to [70, 200] and S belongs to [0.17, 1], the green area of crop leaves can be roughly represented. Using the HSI color gamut, the above areas are erased to achieve the purpose of filtering the chlorophyll [15]. Then the gray values of all pixels are traversed to maximize the inter-class variance, and the obtained *T* is the required threshold. The color interval of each pixel is determined by the solved threshold value to realize the segmentation of pixel values. The final disease spot segmentation result can be obtained by merging multiple segmentation regions.

### 2.5. Extracting the Characteristics of the Diseases and Pests of Citrus Aurantium

Using the feature extraction part in the DCNN, the extraction of the diseases and pests features of Citrus aurantium in the image is realized from the aspects of color and texture.

#### 2.5.1. Color Features

In order to find out the core features of color suitable for Citrus aurantium diseases and pests, according to the color difference of these diseases and pests, multiple characteristic parameters are selected as the color features [16]. We define *r*_*j*_, *g*_*j*_, and *b*_*j*_ as the red, green, and blue components of the *i* th pixel, respectively, and the hue, saturation, and luminance component values of the *i* th pixel of the converted HSI color space are represented as *H*_*i*_, *S*_*i*_, and *I*_*i*_. Then, the extraction of each color feature can be expressed as

(11) $$\begin{array}{c} \left\{\begin{array}{cc} \bar{r}=\frac{1}{N}\sum_{i=1}^{N}r_{i}, & \bar{b}=\frac{1}{N}\sum_{i=1}^{N}b_{i},\;\bar{g}=\frac{1}{N}\sum_{i=1}^{N}g_{i},\\ \bar{H}=\frac{1}{N}\sum_{i=1}^{N}H_{i}, & \bar{S}=\frac{1}{N}\sum_{i=1}^{N}S_{i},\;\bar{I}=\frac{1}{N}\sum_{i=1}^{N}I_{i}, \end{array}\right. \end{array}$$

where $\bar{r}$, $\bar{b}$, $\bar{g}$, $\bar{H}$, $\bar{S}$, and $\bar{I}$ represent the mean values of the red, green, and blue components and the hue, saturation, and luminance components, respectively.

#### 2.5.2. Texture Features

In the field of pattern recognition, texture analysis is a very important work, which involves the details of the image, such as pattern gray distribution, gradient direction, roughness, and so on. Because the disease spots produced by different diseases of Citrus aurantium are always different in texture, the texture feature is selected as the supplement of the color feature, and the two cooperate with each other to avoid the defects of single feature classification. Select the gray level cooccurrence matrix to extract texture features. This method mainly obtains its cooccurrence matrix by calculating the grayscale image and then obtains a series of scalars by calculating the grayscale image to represent the texture information of the image. At any point on the grayscale image, another point is kept a certain distance from the point, and the point pair has a grayscale value [17]. Assuming that the grayscale sequence of the image is, then the grayscale values of the two pixels have a total of combinations. On the entire grayscale image, count the number of occurrences of each to obtain a statistical matrix of, which is called the grayscale co-occurrence matrix, and then normalize this matrix to obtain the joint probability matrix of the grayscale distribution of the image. Based on this model, energy, entropy, and moment of inertia are calculated as texture feature quantities, respectively.

By integrating the extraction results of color features and texture features in the collected images of Citrus aurantium diseases and pests, the extraction results of comprehensive features of Citrus aurantium diseases and pests can be obtained.

### 2.6. Identifying Citrus Aurantium Diseases and Pests

In the DCNN constructed in this study, the extracted image features are resubstituted. Through network training and iteration, the classification results can be obtained, that is, the function of identifying Citrus aurantium diseases and pests.

The training process of DCNN can be divided into two stages: forward propagation and back propagation. Forward propagation is to obtain the calculation result to be inferred, and back propagation is to update the parameters according to the gradient calculated by the loss. The algorithm calculates the output and loss of each layer through forward propagation of the network and calculates the gradient of the network through back propagation [18]. The parameters are then gradient updated according to the stochastic gradient descent algorithm. After continuous learning to make the final loss meet the accuracy requirements, the parameter values of each layer of the network can be retained without reinitialization the next time the network is used [19].

For the identification of Citrus aurantium diseases and pests, it is necessary to set a comparison standard to clarify the color and texture differences between normal Citrus aurantium and abnormal ones, and to set a specific identification and comparison standard map according to the severity of the disease and pest [20]. Then, the similarity between the standard Citrus aurantium image features in the database and the pest features extracted from the DCNN is calculated to realize the matching of pest features. The calculation formula is given by

(12) $$\begin{array}{c} \text{Sim}\left(F_{x},F_{y}\right)={\left(\sum_{i=1}^{n}{\left|F_{x_{i}}-F_{y_{i}}\right|}^{p}\right)}^{1/p}, \end{array}$$

where *F*_*x*_ and *F*_*y*_ represent the extracted image features and standard Citrus aurantium diseases and pests features in the database, respectively, and the variable *p* takes a constant value. By setting the similarity threshold value and combining the results in equation (12), we can obtain the class and severity degree of Citrus aurantium diseases and pests, that is, to obtain the identification results of Citrus aurantium diseases and pests.

## 3. Results and Analysis

In order to test the performance of the proposed identification method based on DCNN, the following test experiments are designed.

In the experiment, the traditional method based on machine vision (the method in reference [4]) and the method based on spatial pyramid pooling (the method in reference [5]) were used for comparison, including traditional recognition methods and algorithm optimization methods. The recognition rates of different methods were calculated and compared in the same experimental environment.

### 3.1. Selecting the Citrus Aurantium Sample Dataset

Three different experimental datasets were employed in the experiment, namely, MalayaKew dataset, P1antVillage dataset, and AES-CD2020 dataset. These MalayaKew leaf datasets were from the Royal Botanic Gardens in Kew, UK, and contain two subsets, MK-D1 and MK-D2, with a total of 44 classes. MK-D1 is a leaf image dataset that performs multi-angle rotation expansion on the collected images to form a training set with 2282 samples and a test set with 528 samples. MK-D2 is an image set formed by local cropping and multi-angle rotation expansion of all leaves in MK-D1. The training set of MK-D2 has 788 images per class, and the testing set has 200 images per class. The P1antVillage dataset is a set of images that contain the health and disease of a variety of plants. There are 38 classes of healthy and diseased images related to crop diseases, more than 50,000 images, and the number of each class of images is uneven.

This study selected 10,478 leaf images of Citrus aurantium collected by P1antVillage, including images of healthy leaves and 5 classes of diseased leaves. The above two experimental sample datasets mainly provide comparison for the experiment. The AES-CD2020 dataset is a dataset composed of images shot on-site. The images in the AES-CD2020 dataset have different sizes, shooting angles, backgrounds, and lighting, etc. The environmental conditions are shown in Figure 4.

All the images in the experimental training set are equally divided into 5 groups, with 200 images in each group. The specific composition of each group of images is shown in Table 1. The data in Table 1 is set as the identification standard data of the experiment.

### 3.2. Experimental Environment

The experiments were designed using the Caffe framework. Caffe is an open source tool for deep learning with CNNs. Caffe supports the languages of are C++ and CUDA and provides MATLAB, Python interfaces, and command lines, where the set_mode interface can be used to switch between CPU and GPU. The selected Citrus aurantium sample dataset was preprocessed to generate a database format. First, Caffe was used to read the data, and then training was performed. Net completed the initialization of the network layer, and Solver was used to control the model training process. During the training process and at the end of the training, several trained models were saved. Through the configuration of the experimental environment, it is ensured that the constructed DCNN could run normally in the experimental environment.

### 3.3. Testing Process and Results Analysis of the Identification Methods

The recognition rate is used as the indicator for evaluating the algorithm performance. It can be directly obtained by calculating the ratio of the number of correctly identified samples to the total number of all identified samples. The prepared experimental sample data was imported into the experimental environment, and the resolution of the data sample was adjusted to 600 × 600. At the same time, the three methods for comparison were imported into the experimental environment in the form of program codes. The identification results were obtained by retrieving data samples.

By comparing the output recognition results with the dataset in Table 1, the results of recognition rate can be obtained, as shown in Table 2.

According to the data in Table 2, the average recognition rates of the methods in [4] and [5] are 87.0% and 91.5%, respectively. By comparison, the DCNN-based identification method proposed in this research shows an average recognition rate of 98.9%, indicating its best performance.

## 4. Conclusions

In order to achieve effective control and prevention of Citrus aurantium diseases and pests, this study designs a DCNN-based method for identifying Citrus aurantium diseases and pests. The method uses the relevant hardware equipment to collect the initial Citrus aurantium leaf images and complete the image preprocessing. The recognition results are obtained through feature matching.

1. In order to verify the effectiveness of the proposed method, relevant experiments have been conducted. The experimental results show that the recognition rate of the proposed method is about 11.9% higher than that of the traditional recognition methods, verifying its high recognition rate.
2. The reason for the high reliability of the proposed method is that it realizes the preprocessing of the initial Citrus aurantium image data through cropping, enhancement, and morphological transformation, etc. This fundamentally avoids the influence of environmental factors on the recognition results.
3. By using the neural network to divide the disease spots of Citrus aurantium images, accurate recognition results are obtained through feature matching. The proposed method can overcome the interference of the external environment to a certain extent and can provide reference data for the prevention and control of Citrus aurantium diseases and pests.

## Figures and Tables

**Figure 1:** Flow chart of the image acquisition of Citrus aurantium diseases and pests.

**Figure 2:** Structure diagram of DCNN.

**Figure 3:** Sigmoid function curve.

**Figure 4:** Schematic diagram of training set samples in the experiment.

**Table 1:** Experimental group setting.

Serial number	1	2	3	4	5
Number of healthy citrus aurantium samples (piece)	66	93	74	85	83
Number of samples of fructus aurantii with leaf blight (piece)	24	17	36	19	27
Leaf spot disease fructus aurantii sample number (piece)	31	25	40	22	25
Powdery mildew fructus aurantii sample quantity (piece)	45	28	11	25	23
Number of samples of thrips citrus (piece)	34	37	39	49	42

**Table 2:** Results of recognition rate.

Serial number		Number of correctly identified samples (piece)	Recognition rate (%)
1	Method of reference [4]	175	87.5
2		173	86.5
3		171	85.5
4		174	87
5		177	88.5
Average		174.0	87.0

1	Method of reference [5]	182	91
2		184	92
3		185	92.5
4		183	91.5
5		181	90.5
Average		183.0	91.5

1	Method of this paper	196	98
2		199	99.5
3		198	99
4		199	99.5
5		197	98.5
Average		197.8	98.9

## Data Availability

The labeled dataset used to support the findings of this study is available from the corresponding author upon request.
